# A Retrospective Analysis of Metagenomic Next Generation Sequencing (mNGS) of Cerebrospinal Fluid from Patients with Suspected Encephalitis or Meningitis Infections

**DOI:** 10.1155/2022/5641609

**Published:** 2022-04-21

**Authors:** Jina Gu, Lin Chen, Chengjun Zeng, Xiaoyan Yang, Danmei Pan, Hongchao Cao, Qinbin Qian

**Affiliations:** Department of Infectious Medicine HwaMei Hospital, University of Chinese Academy of Sciences, Ningbo 315800, China

## Abstract

We determined the clinical value of metagenomic next-generation sequencing (mNGS) of cerebrospinal fluid (CSF) for the diagnosis of patients with suspected encephalitis or meningitis infection. Clinical data were collected and retrospectively analyzed from patients with suspected cases of encephalitis or meningitis who presented at four hospitals in Ningbo from January 1^st^, 2019 to December 31^st^, 2020. Of a total of 66 suspected cases, 41 (62.12%) were diagnosed with central nervous system infections, which included 18 cases (27.27%) of viral infection, 13 cases (19.70%) of bacterial infection, 3 cases (4.55%) of *Mycobacterium tuberculosis*, 5 cases (7.58%) of fungal infection, and 2 cases (3.03%) of *Rickettsia* infection. From these cases, mNGS identified 25 (37.88%) true-positive cases, 8 (12.12%) false-positive cases, 20 (30.30%) true-negative cases, and 13 (19.70%) false-negative cases. The sensitivity of mNGS was 65.79% with a specificity of 71.43%. The positive rate was higher compared with traditional methods (37.88% vs. 24.39%). The results indicate that mNGS technology is a more sensitive method for detecting suspected infectious encephalitis or meningitis compared with traditional pathogen detection methods.

## 1. Introduction

Infection is one of the main causes of suspected infectious encephalitis or meningitis, which demonstrate high morbidity and mortality rates [1]. The diagnosis of central nervous system (CNS) infections is carried out primarily by fluid smear microscopy, pathogen culture, antigen-antibody detection, and polymerase chain reaction (PCR) testing. However, current comprehensive conventional diagnostic technologies can only identify approximately half of all CNS pathogens [2, 3].

Metagenomic next-generation sequencing (mNGS) technology can be used to detect DNA or RNA sequences in biological samples by shotgun sequencing. This novel technique may be used to analyze the genome, transcriptome, and microbiome in patient samples to obtain information regarding pathogenic microorganisms [4]. Recent studies have shown that mNGS may be used to analyze cerebrospinal fluid (CSF) to diagnose CNS infections [5, 6]. However, many disease etiologies detected by mNGS cannot be verified, and some are inconsistent with clinical manifestations. Thus, the etiology of suspected encephalitis or meningitis infections is diverse, and the results of CSF mNGS should be included with standard techniques to improve diagnosis. Therefore, researchers evaluated the results of a clinical study to determine the value of CSF mNGS for patients with suspected infectious encephalitis or meningitis.

## 2. Methods

### 2.1. Research Subjects

This study was a multicenter retrospective analysis of mNGS in CFS samples obtained from patients with suspected infectious encephalitis or meningitis. The study was approved by the ethics committee of Ningbo Hwa Mei Hospital, University of the Chinese Academy of Sciences, and it was approved by the other three participating hospitals. We retrospectively collected clinical data from hospitalized patients at the four hospitals in Ningbo city from January 1^st^, 2019 to December 31^st^, 2020. Patients were screened according to the following inclusion criteria: (i) patients with suspected acute or subacute (course <6 months) encephalitis or meningitis with mNGS analysis of CSF (criteria for suspected encephalitis or meningitis refers to previous studies) [6], and (ii) all patients received a complete diagnosis, and treatment was administered at 1–3 months of follow-up. Patients were excluded from the study based on the following criteria: (i) patients with incomplete data or lost data at follow-up, (ii) patients aged <18 years, (iii) patients with an unknown final diagnosis, (iv) patients in a recovery period after treatment, (v) AIDS patients, (vi) patients with brain trauma or cerebral hemorrhage, and (vii) patients confirmed as presenting with a noninfectious CNS disease before mNGS testing. A total of 85 cases met the inclusion criteria. Based on the exclusion criteria, 19 cases were excluded: 6 because of cerebral hemorrhage, 5 from brain trauma, 1 case in a child, 3 cases because of a lack of information, 1 case because of recovery after treatment, and 3 cases because of failed clinical diagnosis. Finally, 66 patients were included in this study. The process used for the selection of patients is presented in Figure 1.

### 2.2. mNGS Experimental Analysis (mNGS of CSF)

CSF samples were collected by standard aseptic procedures. The samples were frozen and stored at −20°C, and mNGS analysis was performed within 24 hours. RNA and DNA were extracted and randomly amplified (after reverse transcription of the RNA) to generate cDNA molecules for sequencing. Sequencing was performed on the Illumina Nextsep 500/550 or BGISEQ 2000 platforms with an average of 30M reads per sample. The qualified reads were mapped to the human reference genome using the Burrows–Wheeler Aligner to remove human sequences. The remaining reads were aligned to a database for annotation, which included the NCBI microbial genome database (ftp://ftp.ncbi.nlm.nih.gov/genomes/) to detect pathogens [7, 8].

### 2.3. Interpretation of the Traditional Clinical Diagnosis

The diagnosis was confirmed based on clinical manifestations, laboratory and auxiliary examination results, treatment responses, and outcomes. At the end of the follow-up, the diagnosis was made independently by two senior doctors above the level of attending physician, based on the diagnostic criteria of the corresponding guidelines. Cases with different diagnostic opinions were discussed before a definitive diagnosis was made based on the criteria for infectious encephalitis or meningitis used in previous studies [9–12]. The reliability of the final diagnosis was divided into three categories: (i) confirmed cases with evidence of etiology, serology, or pathology except for mNGS; (ii) diagnosis based on clinical manifestations meeting the corresponding diagnostic criteria, the indications of effective treatments, with similar diseases were excluded; and (iii) cases in which the diagnosis was not determined (these cases were excluded).

### 2.4. Interpretation of mNGS Results

CSF samples were analyzed by mNGS using the services of several mNGS detection companies. Currently, no unified standard exists for mNGS analysis of CSF, and so, the suspected pathogens and human colonizing bacteria in the report were removed. If the pathogen detected was consistent with the clinical manifestations and confirmed by traditional microbiological detection methods or consistent with clinical manifestations and no other CNS diseases were evident during follow-up, the cases were considered true positives. False positives were defined as cases in which the detected pathogen was inconsistent with the clinical manifestations or specific treatment, and cases in which other detection methods confirmed noninfectious CNS diseases. True-negative cases were defined if no pathogen was detected by mNGS and the clinical diagnosis was noninfectious encephalitis or meningitis with no evidence of infectious CNS diseases. False-negative cases were defined if no pathogens were detected by mNGS, when the traditional etiology test was positive, which was consistent with clinical manifestations, or when the clinical manifestations were consistent with infectious encephalitis or meningitis. Also, false negatives included cases in which specific antimicrobial treatment was effective and patients showed no evidence of noninfectious CNS disease during follow-up [13]. The results were reviewed by two clinicians and one microbiologist, and controversial cases were excluded. For example, mNGS detection shows mycobacterium tuberculosis complex with a species-specific read number (SSRN) of 7, whereas traditional methods for microbiological detection of CSF are negative, including Xpert MTB/RIF, acid fast stain, and tuberculosis culture. However, if the clinical manifestations, routine biochemical tests of CSF, and head MRI of the patient are consistent with tuberculous meningitis, and the antituberculosis treatment is effective, the case would be judged by the mNGS results as a true positive.

### 2.5. Statistical Analysis

All the data were checked and processed using Microsoft Excel. SPSS18.0 software was used for statistical analysis. The counted data are presented as the rate or constituent ratio and were analyzed by a chi-square test. *P* values <0.05 were considered statistically significant. The measured data were described by $\bar{X}$ ± *s* or median values (interquartile interval) and analyzed using a *t*-test with a threshold value of *P* < 0.05 for statistical significance.

## 3. Results

### 3.1. Clinical Data

A total of 66 patients were included in this study consisting of 37 males and 29 females with an average age of 48.53 ± 19.17 years. The enrolled patients were from the Department of Infectious Diseases, the Neurology Department, the ICU, the Hematology Department, and other departments. Next, DNA mNGS was performed on 58 patient samples (87.88%), whereas both DNA and RNA mNGS were performed in only 9 patients (13.64%). Fifty-eight patients (87.88%) exhibited a fever, and 35 patients exhibited a headache (Table 1).

### 3.2. Results of mNGS of CSF Samples

A total of 41 cases (62.12%) were finally diagnosed with CNS infection, of which 18 cases (27.27%) were infected with viruses, 13 cases (19.70%) with bacteria, 3 cases (4.55%) with *Mycobacterium tuberculosis*, 5 cases (7.58%) with fungi, and 2 cases (3.03%) with *Rickettsia*. 25 cases (37.88%) of non-CNS infection were found including 6 cases (9.09%) of autoimmune encephalitis, 4 cases (6.06%) of vasculitis, and 4 cases (6.06%) of intracranial tumor infiltration. Of the 66 patients, 33 (50.00%) were confirmed. As PCR for multiple viruses at local hospitals could not be carried out, 10 cases (24.39%) were diagnosed with confirmed CNS infections, and 31 cases (75.61%) were only diagnosed clinically.

Of the 66 samples, 33 (50.00%) were positive, 25 (37.88%) were true-positive, and 8 (12.12%) were false-positive. Twenty cases (30.30%) were true negatives, and 13 cases (19.70%) were false negatives. The positive predictive value (PPV), negative predictive value (NPV), and sensitivity and specificity were calculated to evaluate the value of CSF mNGS. Using a clinical diagnosis as the gold standard, mNGS of CSF demonstrated a sensitivity of 65.79%, a specificity of 71.43%, a PPV of 75.76%, and a NPV of 60.61% (Table 2). Of the 41 patients who were finally diagnosed with infectious encephalitis or meningitis, 25 (60.98%) cases were true positives based on mNGS, whereas 10 (24.39%) cases were positive based on traditional microbiological methods. Of the 13 patients who were finally diagnosed with bacterial meningitis, 8 cases (61.54%) were true positives based on mNGS, including 2 cases of *Klebsiella pneumoniae*, 1 case of *Streptococcus pneumoniae*, 1 case of *Streptococcus mitis,* and 4 cases of *Staphylococcus.* Five cases (38.46%) were positive based on traditional microbiological tests, including 1 case of *Streptococcus constellatus*, 1 case of Nocardia, 1 case of *Klebsiella pneumoniae,* and 2 cases of Staphylococcus aureus. Two cases were both positive based on mNGS and traditional microbiological tests, including 1 case of *Staphylococcus aureus* and 1 case of *Klebsiella pneumoniae* (Table 3). Of the 18 patients who were finally diagnosed with viral encephalitis or meningitis, 8 (44.44%) were positive based on mNGS, whereas only 2 (11.11%) cases were positive based on conventional microbiological tests (Table 4). Of the 5 patients who were finally diagnosed with fungal meningitis, 5 (100%) were positive based on mNGS, including 1 case of *Candida albicans*, 1 case of *Cryptococcus*, 1 case of *Candida parapsilosis*, 1 case of *Mucor racemosus,* and 1 case of *Rhizomucor pusillus*. Two (40.00%) cases were positive based on traditional microbiological tests, including 1 case of *Cryptococcus* and 1 case of *Candida albicans*. Of the 3 patients who were finally diagnosed with Tuberculous meningitis, two (66.7%) were positive based on mNGS, whereas 1 case was confirmed by the Xpert MTB/RIF. Also, we found 2 cases (3.03%) with *Rickettsia*. Although we did not have technology to confirm it, after specific clinical treatment, the patient was cured. Interestingly, in patients with noninfectious encephalitis or meningitis, 5 patients tested positive by CSF mNGS, including viruses and multiple bacteria, which we considered false positives, although the possibility of autoimmune encephalitis after viral infection could not be ruled out. The details of the true-positive cases based on the mNGS results are shown in Figure 2.

## 4. Discussion

In this study, we retrospectively analyzed clinical data from multiple centers and reported on 66 suspected cases of infectious encephalitis or meningitis. CSF samples were collected from several departments including infection, neurology, hematology, ICU, and rheumatology and immunology. Suspected cases of infectious encephalitis or meningitis were identified in all departments. The clinical manifestations and laboratory examinations for the patients were similar; however, the causes of infection varied. The number of noninfectious cases was 37.88%.

For noninfectious CNS diseases, diagnosis may be confirmed by assessing autoimmune brain antibodies and CSF pathology. In 41 infectious cases, only 10 cases (24.39%) were confirmed, with the remaining 31 cases (75.61%) being diagnosed only by clinical manifestations, cerebrospinal fluid examination results, and imaging. mNGS of CSF samples exhibited a specificity of 71.43% and a NPV of 60.61%, indicating that mNGS can distinguish infections of the CNS from noninfectious diseases.

Twenty-five cases identified by mNGS of CSF were true positives, with a positivity rate of 37.88%, which was similar to the results of Fan et al. [6]. With respect to bacterial meningitis, we excluded patients with cerebral hemorrhage and postoperative infection following brain trauma; thus, the included patients consisted mainly of those with community-acquired bacterial encephalitis. A previous study [14] showed that *Streptococcus pneumoniae, Neisseria meningitidis,* and *Listeria monocytogenes* are the most common pathogens that cause community-acquired bacterial meningitis. In the present study, *Staphylococcus aureus* and *Klebsiella pneumoniae* were also common. For bacterial meningitis, 8 cases (61.54%) were positive based on mNGS, and the reporting time was less than 48 hours. Five cases (38.46%) were positive based on traditional microbiological tests. Three cases were positive based on cultures, but they were negative by mNGS analysis, including 1 case of *Streptococcus constellatus*, 1 case of Nocardia, and 1 case of *Klebsiella pneumoniae*. The diagnosis of the Nocardia patient was confirmed by a positive abscess fluid culture. The observation of positive results based on cultures and negative results by mNGS may be related to the large quantity of sequencing data in the samples [15] and the use of antimicrobial agents before sequencing.

Currently, few viral detection methods are routinely used in Chinese hospitals. Among the 18 patients who were diagnosed with viral encephalitis or meningitis, only 2 (11.11%) presented with a confirmed diagnosis, and 8 (44.44%) patients were positive based on mNGS. Of the DNA viruses that cause CNS infection, the varicella zoster virus is common. This finding differs from previous reports [16], but it is consistent with domestic reports [17]. The frequency of varicella zoster virus cases may be related to the area from which the patients were sampled, but these findings require further validation. It should also be noted that only DNA sequences were detected in 57 cases (86.36%), whereas RNA viruses were not detected.

The advantages of mNGS technology are primarily reflected in the detection of rare or even unknown pathogens, which is difficult to accomplish by targeted detection. For example, *Pseudorabies* virus encephalitis can be diagnosed in CSF using mNGS technology, and *Pseudorabies* virus can cause severe viral encephalitis in humans [18]. In the present study, two patients were found to be present with *Rickettsia felis* infection, one of whom was admitted to the ICU and quickly improved after treatment. However, the other patient exhibited a fever and improved after chloramphenicol treatment. Currently, no reported cases of *Rickettsia felis* intracranial infection have been found in China, and foreign reports are also rare [19, 20].

Eight cases (12.12%) were found to be false positives based on mNGS analysis of CSF. Multiple bacteria and fungi were detected in 2 cases of viral encephalitis or meningitis and 3 cases of noninfectious diseases in which the traditional pathogenic test was negative. Contamination of samples was considered, including *Staphylococcus hominis, Stenotrophomonas maltophilia, Schizophyllum, Enterococcus flavus, and Enterococcus casseliflavus.* Epstein–Barr virus (EBV) was detected in 1 case of autoimmune encephalitis and 1 case of tuberculous meningitis. Human polyomavirus type 5 was detected in 1 case of intracranial infiltration of leukemia. Although the reads per million mapped readers (RPM) for these viruses reached the standard of RPM ≥3, which is recognized in other studies [5, 6], we still considered these cases as false positives.

## 5. Conclusion

In conclusion, mNGS analysis of CSF requires further development and validation before routine use, although we demonstrated that it exhibits utility for the diagnosis of patients with suspected infectious encephalitis or meningitis. This diagnostic approach facilitates early diagnosis and treatment and enables the identification of emerging infectious pathogens and infectious diseases. In clinical practice, combining mNGS with traditional microbial detection methods may improve the diagnosis and treatment of neuroinfectious diseases; however, this process requires further optimization. Our data may be subject to diagnosis bias because it was collected from a retrospective study and confirmation of cases by PCR cannot be carried out routinely. In the future, prospective studies are needed to evaluate the utility of mNGS analysis of CSF in clinically suspected cases of infectious encephalitis or meningitis.

## Figures and Tables

**Figure 1:** Flowchart of patient enrollment and exclusion.

**Figure 2:** 25 cases of true-positive results.

**Table 1:** Clinical data of 66 patients included in the study.

Factors		Number of cases	Percentage (%)
Sex	Male	37	56.06
	Female	29	43.94
Age (years; mean ± SD)	48.53 ± 19.17		
Department	Hematology department	11	16.67
	ICU	11	16.67
	Department of infection	26	39.39
	Neurology department	13	19.7
	Other departments	5	7.58
Type of mNGS	Single DNA sequencing	57	86.36
	Both DNA + RNA sequencing	9	13.64
Underlying disease	Malignant tumor	11	16.67
	Immunosuppression	17	25.76
Clinical manifestation	Fever	58	87.88
	Headache	35	53.03
	Change of consciousness or personality	17	25.76
	Epilepsy	10	15.15
	Neck rigidity	11	16.67
Outcome	Admission to ICU	13	19.7
	Death	11	16.67

**Table 2:** mNGS results and clinical diagnosis of CSF data.

Clinical diagnosis	mNGS				
	True positive	False positive	True negative	False negative	Total
Bacterial meningitis	8	0	0	5	13
Viral encephalitis/meningitis	8	2	0	8	18
Tuberculous meningitis	2	1	0	0	3
Fungal meningitis	5	0	0	0	5
Rickettsia encephalitis	2	0	0	0	2
Noninfectious	0	5	20	0	25
Total	25	8	20	13	

**Table 3:** Comparison of CSF mNGS and CSF culture results in 13 patients with bacterial meningitis.

mNGS	Traditional methods for microbiological detection of CSF		
	Positive	Negative	Total
Positive	2	6	8
Negative	3	2	5
Total	5	8	

**Table 4:** Comparison of CSF mNGS and traditional microbiological detection results for 18 patients with viral encephalitis or meningitis.

mNGS	Traditional methods for microbiological detection of CSF		
	Positive	Negative	Total
Positive	2	6	8
Negative	0	10	10
Total	2	16	

## Data Availability

The data used to support the findings of this study are available from the corresponding author upon request.
